# Rosuvastatin suppresses platelet-derived growth factor-BB-induced vascular smooth muscle cell proliferation and migration via the MAPK signaling pathway

**DOI:** 10.3892/etm.2013.1265

**Published:** 2013-08-20

**Authors:** JIANTING GAN, PING LI, ZHENGDONG WANG, JIAN CHEN, XIANGWEN LIANG, MING LIU, WENCHAO XIE, RUIXING YIN, FENG HUANG

**Affiliations:** 1 Department of Cardiology, Sixth Affiliated Hospital of Guangxi Medical University, Yulin, Guangxi 537000;; 2 Department of Cardiology, First Affiliated Hospital of Guangxi Medical University, Nanning, Guangxi 530021, P.R. China

**Keywords:** rosuvastatin, vascular smooth muscle cell, platelet-derived growth factor, proliferation, migration, mitogen-activated protein kinase

## Abstract

An imbalance in the proliferation and migration of vascular smooth muscle cells (VSMCs) is significant in the onset and progression of vascular diseases, including arteriosclerosis and restenosis subsequent to vein grafting or coronary intervention. Rosuvastatin, a selective inhibitor of hydroxymethylglutaryl coenzyme A (HMG-CoA) reductase, has pharmacological properties including the ability to reduce low-density lipoprotein-cholesterol (LDL-C) and very low-density lipoprotein-cholesterol (VLDL-C) levels, slow atherosclerosis progression and improve coronary heart disease outcomes. However, little is known concerning the molecular mechanism by which rosuvastatin affects vascular cell dynamics. In this study, we studied the inhibitory role of rosuvastatin on platelet-derived growth factor-BB (PDGF-BB)-induced VSMC proliferation and migration, as well as the molecular mechanisms involved. MTT data showed that rosuvastatin markedly inhibited the proliferation of PDGF-BB-induced VSMCs in a time-dependent manner. VSMCs are able to dedifferentiate into a proliferative phenotype in response to PDGF-BB stimulation; however, rosuvastatin effectively attenuated this phenotype switching. Moreover, we also showed that rosuvastatin significantly suppressed PDGF-BB-induced VSMC migration, which may be a result of its inhibitory effect on the protein expression of matrix metalloproteinase-2 (MMP2) and MMP9. Investigation into the molecular mechanisms involved revealed that rosuvastatin inhibited the mitogen-activated protein kinase (MAPK) signaling pathway by downregulating extracellular signal-regulated kinase (ERK) and p38 MAPK, although the phosphorylation level of c-Jun N-terminal kinase (c-JNK) was not altered following rosuvastatin treatment. In conclusion, the present study showed that rosuvastatin suppressed PDGF-BB-induced VSMC proliferation and migration, indicating that rosuvastatin has the potential to become a promising therapeutic agent for the treatment of atherosclerosis and restenosis.

## Introduction

The unbalanced proliferation of vascular smooth muscle cells (VSMCs) acts as a critical factor in the initiation and progression of vascular diseases, such as restenosis and arteriosclerosis, subsequent to coronary intervention or vein grafting (1,2). Therefore, antiproliferative agents for VSMCs may serve as effective strategies for attenuating proliferative vascular diseases, as well as for reducing the incidence of cardiovascular complications, including bypass graft failure and in-stent restenosis (3,4).

It has been well established that during the repair of vascular injury, multiple cytokines and growth factors are released that stimulate vascular cell proliferation (5–7). For example, following angioplasty, the upregulated production of platelet-derived growth factor (PDGF) initiates proliferation-related signaling pathways to stimulate VSMC proliferation in response to vascular injury (8,9). As a result, developing effective agents to suppress the PDGF-induced abnormal proliferation of vascular cells shows promise for improving the efficacy of cardiovascular surgery.

Hydroxymethylglutaryl coenzyme A (HMG-CoA) reductase catalyzes the conversion of 3-hydroxy-3-methylglutaryl CoA to mevalonate, a precursor of cholesterol (10). As a result, HMG-CoA reductase inhibitors, such as statins, may be utilized for lowering cholesterol. Among all statins, rosuvastatin is a selective HMG-CoA reductase inhibitor, the main action site of which is the liver, the target organ for lowering cholesterol (11). Rosuvastatin increases the number of hepatic cell surface receptors for low-density lipoprotein-cholesterol (LDL-C), promotes the absorption and catabolism of LDL-C and inhibits the synthesis of very low-density lipoprotein-cholesterol (VLDL-C), thereby reducing total VLDL-C and LDL-C levels. Moreover, rosuvastatin is also able to reduce plasma triglycerides and increase high-density lipoprotein-cholesterol (HDL-C) levels (12). It has been shown that rosuvastatin is able to slow atherosclerosis progression and improve coronary heart disease outcomes (11); however, the molecular mechanism behind the action of rosuvastatin on vascular cell dynamics has not been fully elucidated.

Therefore, this study aimed to investigate whether rosuvastatin was able to inhibit PDGF-BB-stimulated VSMC proliferation and migration, as well as the associated molecular mechanism.

## Materials and methods

### Materials and agents

Rosuvastatin was obtained from AstraZeneca (London, UK). Recombinant mouse PDGF-BB was purchased from Supbio Company (Changsha, China). DMSO and MTT were obtained from Sigma-Aldrich (St. Louis, MO, USA), while antibodies for smooth muscle-α-actin (SMA), smoothelin, desmin, phospho-extracellular signal-regulated kinase 1/2 (ERK1/2), ERK, phospho-p38, p38, phospho-c-Jun N-terminal kinase (JNK), JNK, matrix metalloproteinase-2 (MMP2), MMP9 and glyceraldehyde 3-phosphate dehydrogenase (GAPDH) were purchased from Santa Cruz Biotechnology, Inc. (Santa Cruz, CA, USA).

### Cell culture

VSMCs were isolated from the thoracic aortas of Sprague Dawley rats, and cultured in DMEM/F12 medium containing 10% fetal bovine serum (FBS). VSMCs of passage five were used in this study.

### MTT assay

VSMCs were cultured to 70% confluence and serum-starved for 24 h. In the experimental group, cells were treated with rosuvastatin (10 *μ*M) and PDGF-BB (20 ng/ml) for 6, 12, 24 and 48 h. In the control group, cells were cultured without any treatment. In the negative control (NC) group, cells were treated only with PDGF-BB (20 ng/ml) for 6, 12, 24 and 48 h. Following treatment, an MTT assay was used to examine the viability of the cells in all groups. Cells were plated at a density of 10^4^/well, and incubated at 37°C with 5% CO_2_ for 3 h, subsequent to adding MTT (Promega, Madison, WI, USA) to the medium at a final concentration of 0.5 *μ*g/ml. The medium was then removed and 100 *μ*l DMSO was added. The plate was gently rotated on an orbital shaker for 10 min to completely dissolve the precipitation. A microplate reader (Bio-Rad, Hercules, CA, USA) was used to determine the absorbance at 570 nm.

### Cell migration assay

For all groups, migration was measured in 24-well Transwell chambers (Chemicon, Temecula, CA, USA). In the control group, cells were cultured without any treatment. In the NC group, cells were cultured following the addition of PDGF-BB (20 ng/ml). In the experimental group, cells were cultured with rosuvastatin (10 *μ*M) and PDGF-BB (20 ng/ml). Subsequent to 24 h incubation at 37°C with 5% CO_2_, the migrated cells were stained and counted.

### Western blot analysis

In the control group, the cells were cultured without any treatment. In the NC group, cells were cultured following the addition of PDGF-BB (20 ng/ml) for 48 h. In the experimental group, cells were cultured with rosuvastatin (10 *μ*M) and PDGF-BB (20 ng/ml) for 48 h. Cold radio-immunoprecipitation assay (RIPA) lysis buffer was used to solubilize the cells. Protein was separated with 5% sodium dodecyl sulfate-polyacrylamide gel electrophoresis (SDS-PAGE) and transferred to a polyvinylidene difluoride (PVDF) membrane. The membranes were blocked in 5% non-fat dried milk in phosphate-buffered saline (PBS) overnight, prior to being incubated with specific primary antibodies (Santa Cruz Biotechnology, Inc.) for 3 h. Primary antibodies for SMA, smoothelin, desmin, p-ERK1/2, ERK, phospho-p38, p38, phospho-c-JNK, JNK, MMP2, MMP9 and GAPDH were used. All antibodies were mouse monoclonal antibodies bought from Santa Cruz Biotechnology, Inc. (Santa Cruz, CA, USA). Following incubation with rabbit anti-mouse secondary antibody (Santa Cruz Biotechnology, Inc.), immune complexes were detected using an enhanced chemiluminescence (ECL) Western Blotting Substrate kit (Biovision, San Francisco, CA, USA).

### Statistical analysis

Data are expressed as the mean ± standard deviation (SD) and analyzed using one-way analysis of variance (ANOVA). All analyses were performed using SPSS 17.0 statistical software (SPSS, Inc., Chicago, IL, USA). P<0.05 was considered to indicate a statistically significant difference.

## Results

### Inhibitory effect of rosuvastatin on the proliferation of PDGF-BB-stimulated VSMCs

The effect of rosuvastatin on the proliferation of PDGF-stimulated VSMCs was studied using an MTT assay. As shown in Fig. 1, the cell proliferation rate in the experimental group was significantly reduced in a time-dependent manner when compared with that in the NC group, indicating that rosuvastatin had an inhibitory effect on the cell proliferation of the PDGF-BB-induced VSMCs.

### Inhibitory effect of rosuvastatin on the PDGF-BB-induced phenotype switching of the VSMCs

VSMCs are able to dedifferentiate into a proliferative phenotype in response to vascular injury. Under such conditions, the protein expression of the smooth muscle markers SMA, smoothelin and desmin are decreased. Therefore, we tested whether rosuvastatin was able to regulate the phenotype switching of PDGF-BB-stimulated VSMCs. VSMCs were stimulated with PDGF-BB (20 ng/ml) for 48 h in the presence and absence of 10 *μ*M rosuvastatin. Western blotting data showed that PDGF-BB stimulation reduced the SMA protein expression, indicating the dedifferentiation of the VSMCs into a proliferative phenotype (Fig. 2). However, 10 *μ*M rosuvastatin attenuated this effect, suggesting that rosuvastatin inhibits the switch of PDGF-BB-stimulated VSMCs into a proliferative phenotype.

### Inhibitory effect of rosuvastatin on the PDGF-BB-stimulated migration of VSMCs

We further determined the effect of rosuvastatin on the migration ability of PDGF-BB-stimulated VSMCs. VSMCs were stimulated with PDGF-BB (20 ng/ml) for 48 h in the presence/absence of 10 *μ*M rosuvastatin. As demonstrated in Fig. 3A, PDGF-BB stimulation markedly enhanced the migration of VSMCs when compared with that in the control group without any treatment. However, rosuvastatin significantly inhibited the migration of PDGF-BB-stimulated VSMCs. Western blotting results showed that the protein expression of MMP2 and MMP9 was notably suppressed with rosuvastatin treatment (Fig. 3B).

### Inhibitory effect of rosuvastatin on the mitogen-activated protein kinase (MAPK) signaling pathway activated by PDGF-BB in VSMCs

It has been demonstrated that the MAPK signaling pathway is important in VSMC proliferation in response to PDGF-BB stimulation. Thus, we determined the activity of the MAPK signaling pathway in PDGF-BB-stimulated VSMCs with or without the treatment of rosuvastatin for 48 h. As shown in Fig. 4, western blotting data demonstrated that the phospho-ERK1/2 and phospho-p38 MAPK protein levels in the PDGF-BB-stimulated VSMCs treated with rosuvastatin were significantly lower than those in the PDGF-BB-stimulated VSMCs without rosuvastatin treatment, although the phosphorylation level of c-JNK was not affected. These results indicated that it was likely that rosuvastatin suppressed the proliferation of PDGF-BB-stimulated VSMCs by downregulating the activity of the MAPK signaling pathway.

## Discussion

Rosuvastatin is a selective HMG-CoA reductase inhibitor that has multiple biological activities, which include inhibiting HMG-CoA reductase activity, increasing LDL receptor levels and inhibiting VLDL-C synthesis. As a result, rosuvastatin has been commonly used as an anti-hyperlipidemic therapy. Recently, accumulating evidence has shown that rosuvastatin exhibits anti-arteriosclerotic activity (13). However, the molecular mechanisms of rosuvastatin underlying its actions in vascular diseases, including restenosis and arteriosclerosis, have not been fully elucidated.

Vascular injury leads to the marked upregulation of VSMC proliferation and migration, which further results in neointima formation. In the present study, to the best of our knowledge, we showed for the first time that rosuvastatin effectively suppressed PDGF-BB-stimulated VSMC proliferation and migration *in vitro*, and that these effects may partly be attributed to the downregulation of the activity of the MAPK signaling pathway, as well as the decreased protein expression of MMP2 and MMP9. These data indicate that rosuvastatin may be beneficial in the protection against the neointima formation associated with restenosis and arteriosclerosis subsequent to vein grafting or coronary intervention.

It has been demonstrated that vascular injury may affect VSMC plasticity and lead to the dedifferentiation of VSMCs into a proliferative phenotype (14). Our study showed that PDGF-BB treatment inhibited VSMC proliferation, as well as the protein expression of VSMC markers (smooth muscle markers SMA, smoothelin and desmin), indicating that VSMCs dedifferentiated into a proliferative phenotype. However, rosuvastatin effectively attenuated these alterations, suggesting that rosuvastatin is able to inhibit PDGF-BB-induced VSMC proliferation.

The migration of VSMCs is crucial in the repair of vascular injury, i.e., the development of restenosis and atherosclerotic lesions subsequent to by-pass graft or angioplasty (15), and PDGF-BB has been revealed to have the ability to induce VSMC migration via multiple mechanisms (16–18). In this study, we showed that rosuvastatin effectively inhibited PDGF-BB-induced VSMC migration, accompanied by the decreased protein expression of MMP2 and MMP9. MMP2 and MMP9 are critical enzymes participating in extracellular matrix (ECM) remodeling, as well as cell proliferation and invasion, and are important in cardiovascular diseases (19–22). Thus, we hypothesize that the inhibitory effect of rosuvastatin on PDGF-BB-induced VSMC migration may be partly attributed to its inhibitory effect on the expression of MMP2 and MMP9.

Since the expression levels of MMP2 and MMP9 have been demonstrated to be regulated by the MAPK signaling pathway, which also regulates cell proliferation (23,24), we further determined the phosphorylation levels of three MAPKs in PDGF-BB-stimulated VSMCs with or without rosuvastatin treatment. Although data concerning the phosphorylation of c-JNK revealed no difference, irrespective of rosuvastatin treatment, the phosphorylation levels of ERK1/2 and p38 were significantly upregulated in PDGF-BB-stimulated VSMCs, while rosuvastatin treatment effectively attenuated these effects. This suggests that rosuvastatin had an inhibitory effect on the PDGF-BB-induced MAPK activation in VSMCs. Several other studies have demonstrated that the MAPK signaling pathway participates in the PDGF-BB-induced VSMC proliferation and migration (25,26). Zhao *et al* (25) showed that ERK nuclear translocation was involved in the PDGF-BB-stimulated migration of VSMCs, while Zhu *et al* (26) observed that the phosphorylation of ERK1/2 and p38 was markedly induced following PDGF-BB treatment in VSMCs, which was consistent with our results.

In conclusion, the present study showed for the first time, to the best of our knowledge, that rosuvastatin inhibited PDGF-BB-induced VSMC proliferation and migration, which are critical in neointimal hyperplasia. Moreover, these protective effects were shown to be associated with the cell cycle arrest, the downregulated activity of the MAPK signaling pathway, as well as reductions in the protein expression levels of MMP2 and MMP9. This study indicated that rosuvastatin showed promising effects for preventing the neointima formation associated with arteriosclerosis and restenosis subsequent to vein grafting or coronary intervention.

## Figures and Tables

**Figure 1.** Rosuvastatin inhibited the proliferation of platelet-derived growth factor-BB (PDGF-BB)-stimulated vascular smooth muscle cells (VSMCs). Con, VSMCs were cultured without any treatment; NC, VSMCs were treated only with PDGF-BB (20 ng/ml) for 6, 12, 24 and 48 h; rosuvastatin, VSMCs were treated with rosuvastatin (10 *μ*M) and PDGF-BB (20 ng/ml) for 6, 12, 24 and 48 h. An MTT assay was used to examine the viability of cells in all groups. OD, optical density.

**Figure 2.** Rosuvastatin inhibited the platelet-derived growth factor-BB (PDGF-BB)-induced phenotype switching of vascular smooth muscle cells (VSMCs). Con, VSMCs were cultured without any treatment; NC, VSMCs were treated only with PDGF-BB (20 ng/ml) for 48 h; rosuvastatin, VSMCs were treated with rosuvastatin (10 *μ*M) and PDGF-BB (20 ng/ml) for 48 h. The protein expression levels of the smooth muscle markers smooth muscle-α-actin (SMA), smoothelin and desmin were determined. GAPDH, glyceraldehyde 3-phosphate dehydrogenase.

**Figure 3.** Rosuvastatin suppressed the platelet-derived growth factor-BB (PDGF-BB)-stimulated migration of vascular smooth muscle cells (VSMCs). Con, VSMCs were cultured without any treatment; NC, VSMCs were treated only with PDGF-BB (20 ng/ml) for 48 h; rosuvastatin, VSMCs were treated with rosuvastatin (10 *μ*M) and PDGF-BB (20 ng/ml) for 48 h. (A) Transwell assay was used to determine the migration of VSMCs. (B) Protein expression of matrix metalloproteinase 2 (MMP2) and 9 (MMP9) was determined by western blot analysis. Glyceraldehyde 3-phosphate dehydrogenase (GAPDH) was used as an internal reference. ^**^Significantly different from the NC group (P<0.01).

**Figure 4.** Rosuvastatin inhibited the mitogen-activated protein kinase (MAPK) signaling pathway activated by platelet-derived growth factor-BB (PDGF-BB) in vascular smooth muscle cells (VSMCs). Con, VSMCs were cultured without any treatment; NC, VSMCs were treated only with PDGF-BB (20 ng/ml) for 48 h; rosuvastatin, VSMCs were treated with rosuvastatin (10 *μ*M) and PDGF-BB (20 ng/ml) for 48 h. Western blot analysis was used to determine the protein expression of phospho-extracellular signal-regulated kinase 1/2 (ERK1/2), ERK, phospho-p38, p38, phospho-c-Jun N-terminal kinase (JNK) and JNK. Glyceraldehyde 3-phosphate dehydrogenase (GAPDH) was used as an internal reference.
